The article "Study on Influencing Factors of Frailty in Elderly Patients with Type II Diabetes" was retracted in 2023. Reason: concerns about the peer review.

# Study on Influencing Factors of Frailty in Elderly Patients with Type II Diabetes

**DOI:** 10.1155/2022/7244847

**Published:** 2022-01-29

**Authors:** Yingying Song, Ziwei Lin, Miaomiao Ding, Peipei Yuan, Qianqian Li, Hongli Zhai, Feilong Hu, Lingli Zhang, Junmao Wang

**Affiliations:** ^1^Department of Geriatrics, Bozhou People's Hospital, Bozhou 236800, Anhui Province, China; ^2^General Practice, Bozhou People's Hospital, Bozhou 236800, Anhui Province, China

## Abstract

The purpose of this study was to analyze the influencing factors of frailty in elderly patients with type II diabetes. 332 elderly patients with type II diabetes admitted to our hospital from May 2018 to December 2019 were selected as the study subjects. The degree of frailty was evaluated by the Fried fragility phenotype scale, and the general information and the clinical data of patients were collected by inquiry and questionnaire survey. After that, all the data were analyzed by SPSS 20.0. Univariate analysis showed that there were significant differences in age, medication types, dietary habits, exercise tolerance, exercise capacity, body balance, coordination ability, urinary incontinence, anxiety, etc., in elderly patients with type II diabetes who suffered from different degrees of frailty (*P* < 0.01). In addition, there were significant differences in the presence of coronary heart disease, heart failure, atrial fibrillation, pulmonary diseases, osteoarticular diseases, anemia, and other blood diseases of elderly patients with type II diabetes who suffered from different degrees of frailty (*P* < 0.01). Multiple Logistic regression analyses indicated that weakened exercise tolerance, reduced exercise capacity, atrial fibrillation, anemia, and other blood diseases were the influencing factors of the frailty in elderly patients with type II diabetes. The degree of frailty in elderly patients with diabetes is affected by many factors, such as exercise tolerance, exercise capacity, atrial fibrillation, anemia, and other blood diseases; thus, reasonable intervention should be implemented for elderly patients with type II diabetes according to the influencing factors so as to effectively relieve frailty.

## 1. Introduction

China is one of the countries with a severely aging population and the fastest population growth across the world, which has led to a significant increase in the incidence of many chronic diseases, including diabetes, hypertension, and coronary heart diseases [1,2]. Nowadays, diabetes, mostly affecting middle-aged and elderly patients, is a metabolism-related disease, whose nosogenesis is complex and related to many factors, such as obesity, hypertension, hyperlipidemia, imbalanced diet, and lack of exercise, posing a great threat to peoples' physical health [3, 4]. Further investigation has also revealed that there is a significant correlation between impaired exercise tolerance and reduced neural activity. Nesti et al. [5] have also pointed out that the patients with type II diabetes have significantly decreased exercise tolerance, which may relate to the reduced vascular capacitance. With more and more further studies conducted on diabetes, many reports have pointed out that frailty has a direct relationship with the life quality of elderly patients with diabetes. Frailty is a geriatric syndrome with complex pathogenesis, which can usually be classified into three types according to the degree of frailty in patients, no frailty, mild frailty, and severe frailty, and the frailty is mainly manifested by a significant decline in patients' physical and psychological functions, ultimately triggering adverse outcomes in nervous and motor systems [6, 7]. Several studies have pointed out that the frailty in elderly patients is associated with several factors, including age, exercise capacity, living habits, types of medication taking, physique, and cardiovascular and cerebrovascular diseases. The purpose of the study was to analyze the influencing factors of frailty in elderly patients with type II diabetes. Due to the strictly controlled diet, elderly patients who suffer from cardiovascular and cerebrovascular diseases generally have a poor physique and are easily subject to frailty. The symptoms of frailty are mainly often manifested in physical and psychological aspects. Based on this, 332 elderly patients with type II diabetes were selected in this study to record their degrees of frailty and analyze the influencing factors, with the purpose of providing a reference on relieving the frailty of patients with diabetes.

The article "Study on Influencing Factors of Frailty in Elderly Patients with Type II Diabetes" was retracted in 2023. Reason: concerns about the peer review.

## 2. Subjects and Methods

### 2.1. Study Subjects

332 elderly patients with type II diabetes admitted to our hospital from May 2018 to December 2019 were selected as the study subjects, and their general information are shown in Table 1.

### 2.2. Inclusion Criteria/Exclusion Criteria

Inclusion criteria: (1) Patients aged over 60 years old. (2) Patients were clinically diagnosed with diabetes. (3) Patients were conscious and had no communication disorders. (4) Patients were informed of the purpose and process of the study. (5) Patients voluntarily signed informed consent. (6) Patients had no other malignant diseases that seriously affected this study.

Exclusion criteria: (1) Patients had incomplete clinical data. (2) Patients had type I diabetes. (3) Patients had severe mental illness. (4) Patients could not cooperate with clinical followup. (5) Patients had taken antidepressants or psychiatric medication for a long time.

## 3. Methods

Data collection methods. On the basis of the inclusion and exclusion criteria, the clinical data of the patients were collected through a hospital case management system, and the general information was obtained by inquiry and questionnaire survey. In this study, a total of 340 questionnaires were distributed, and 332 valid questionnaires were returned, with the effective rate reaching up to 97.64%.

General information survey. Demographic sociology such as gender, age, marital status, types of medication taking, and living habits such as dietary habits, drinking history, exercise, and circadian rhythms of the patients were surveyed.

Clinical data survey. Physique-related indexes such as exercise tolerance, exercise capacity, body balance, and coordination ability, and the indexes related to disease symptoms such as urinary incontinence, anxiety, coronary heart diseases, heart failure, atrial fibrillation, pulmonary diseases, osteoarthritis, and anemia of patients were surveyed.

Frailty assessment. The degree of frailty in patients was assessed by the Fried fragility phenotype scale, which consisted of patients' weight loss, weakness, slowed walking speed, decreased grip strength, and physical activity. Grip strength testing was conducted. The grip strength of elderly patients' dominant hands was measured by a hand-held grip dynamometer. During the test, the patients stood upright, with their palms kept inward, and their forearms were parallel to the ground and vertical to the upper arms. Meanwhile, the dynamometer was kept outward. The test was carried out 3 times, and test results were averaged. Each index scored 0 if it was no, and 1 point if it was yes. The total score of 0 was classified as no frailty (grade I), 1 to 2 as mild frailty (grade II), and more than or equal to 3 as severe frailty (grade III).

### 3.1. Statistical Treatment

In this study, data were all analyzed by SPSS 21.0, and enumeration data were tested by the *X*^2^ test. Multiple logistic regression analyses were performed to analyze the influencing factors of the frailty in patients with diabetes. The differences had statistical significance when *P* < 0.05.

## 4. Results

### 4.1. Univariate Analysis of Frailty in Elderly Patients with Type II Diabetes

Univariate analysis of relevant factors such as living habits of elderly patients with type II diabetes was conducted, as shown in Table 2. There were significant differences in the age, types of medication taking, dietary habits, and the exercise of elderly patients with type II diabetes who suffered from different degrees of frailty (*P* < 0.01).

The article "Study on Influencing Factors of Frailty in Elderly Patients with Type II Diabetes" was retracted in 2023. Reason: concerns about the peer review.

Univariate analysis of relevant factors such as physique including exercise tolerance, exercise capacity, body balance, coordination ability, urinary incontinence, and anxiety was conducted, as shown in Table 3. There were significant differences in the exercise tolerance, exercise capacity, body balance, coordination ability, urinary incontinence, and anxiety of elderly patients with diabetes who suffered from different degrees of frailty (*P* < 0.01).

Univariate analysis of the factors related to cardiovascular diseases including coronary heart diseases, heart failure, and atrial fibrillation of elderly patients with type II diabetes was carried out, as shown in Table 4. There were significant differences in the presence of coronary heart disease, heart failure, atrial fibrillation, and other diseases of elderly patients with type II diabetes who suffered from different degrees of frailty (*P* < 0.01).

Univariate analysis of the factors related to other diseases including pulmonary diseases, osteoarticular diseases, anemia, and other blood diseases of elderly patients with type II diabetes was conducted, as shown in Table 5. There were significant differences in pulmonary diseases, osteoarticular diseases, anemia, and other blood diseases of elderly patients with type II diabetes who suffered from different degrees of frailty (*P* < 0.01).

### 4.2. Multiple Logistic Regression Analysis of Influencing Factors of Frailty in Elderly Patients with Type II Diabetes

The results of multiple logistic regression analysis of the influencing factors of frailty in elderly patients with type II diabetes showed that the presence of exercise intolerance, weakened exercise capacity, atrial fibrillation, anemia, and other blood diseases were the influencing factors of frailty in elderly patients with type II diabetes (*P* < 0.01), as shown in Table 6.

## 5. Discussion

Type II diabetes is one of the major diseases threatening elderly patients' physical health and often causes several complications affecting the heart and cerebral vessels, livers, kidneys, and the integumentary system [8, 9]. Due to the strictly controlled diet, elderly patients who suffer from cardiovascular and cerebrovascular diseases generally have a poor physique and are easily subject to frailty. The symptoms of frailty are mainly often manifested in physical and psychological aspects. For example, patients are presented with negative emotions, cognitive impairment, weakness, and low activity, which seriously affect their daily life and weaken the normal body function [10, 11]. However, the nosogenesis of frailty in elderly patients with type II diabetes is complicated and related to several factors. Based on this, this study analyzed the causes of frailty in terms of age and living habits, patients' physique, cardiovascular diseases, and other diseases to provide a valid reference for the treatment of frailty in elderly patients with type II diabetes.

The article "Study on Influencing Factors of Frailty in Elderly Patients with Type II Diabetes" was retracted in 2023. Reason: concerns about the peer review.

Our study demonstrated that exercise intolerance was significantly associated with frailty in elderly patients with type II diabetes. Exercise tolerance is one of the important indexes that can reflect people's physique, and patients with frailty can easily suffer from exercise intolerance [12]. Ishihara et al. [13] have found that compared with normal people, the patients with type II diabetes mostly lack lower limb strength during exercise and have significantly weakened activity in autonomic nerves, sympathetic nerves, and parasympathetic nerves. Nowadays, diabetes, mostly affecting middle-aged and elderly patients, is a metabolism-related disease, whose nosogenesis is complex and related to many factors, such as obesity, hypertension, hyperlipidemia, imbalanced diet, and lack of exercise, posing a great threat to peoples' physical health [3,4]. Further investigation has also revealed that there is a significant correlation between impaired exercise tolerance and reduced neural activity. Nesti et al. [5] have also pointed out that the patients with type II diabetes have significantly decreased exercise tolerance, which may relate to the reduced vascular capacitance. Exercise capacity is an important index for measuring patients' body function and psychological reconciliatory ability. Our study results showed a significant correlation between weakened exercise capacity and frailty in elderly patients with type II diabetes. Machii et al. [14] have demonstrated that patients with type II diabetes often have significantly reduced exercise capacity, which is manifested by slow gait speed during walking speed, decreased grip strength, and muscular atrophy. Kuziemski et al. [15] have reported that the patients with frailty mainly have weakened pulmonary function and weakness during walking, adversely affecting their exercise capacity. In this study, the degree of frailty in elderly patients with type II diabetes was significantly correlated with the presence of anemia and blood diseases. These studies are relatively in line with the conclusions of our study that the elderly patients generally have a poor physique, and some of them even have difficulty in moving, thus leading to their less exercise and seriously affecting their physical health [16–18]. All of these studies suggest that exercise intolerance in patients with type II diabetes can reflect the degree of frailty to a certain extent, which has great significance in the timely diagnosis and treatment of this disease. Therefore, in routine nursing care, in addition to strict monitoring of patients in terms of diet as well as insulin levels, suitable protocols need to be developed for their daily exercise interventions so as to gradually improve patients' exercise capacity and exercise intolerance under the premise of ensuring safety, ultimately maintaining their normal body function and relieving frailty. Studies have shown that anemia and other blood diseases are the main causes of patients' frailty, and the patients with anemia are mostly subject to poor blood circulation, blood insufficiency, and other symptoms, while all of these conditions can affect the blood supply to brains, which further damages patients' neurons, thereby leading to the symptoms of frailty [19, 20]. Palmer et al. [21] have retrospectively analyzed 19 studies and concluded that anemia was significantly associated with frailty, and the incidence of frailty in elderly patients with anemia was twice more than that of normal people, suggesting that anemia is one of the key factors leading to frailty in elderly patients with type II diabetes. The intake of sugar and nutrients is usually tightly controlled in elderly patients with type II diabetes, which leads to their vulnerability to anemia. Based on this, in the daily nursing care of elderly patients, some vitamins and trace elements such as iron and zinc should be appropriately supplemented on the basis of controlling energy intake, thereby improving anemia to relieve frailty. Atrial fibrillation, as a persistent and frequent arrhythmia in elderly patients, is often associated with factors such as coronary heart diseases, hypertension, and heart failure, and clinically, the patients often present with rapid heart rate, reduced cardiac systolic function, and heartbeat frequency. [22–24]. Our study results showed that there was a close association between the presence of atrial fibrillation and the degree of frailty in elderly patients with diabetes. Slawuta et al. [25] have found the retrospective analysis of clinical data from 158 elderly patients with diabetes that compared with the patients in the normal group, those with frailty mostly suffered from arrhythmia and atrial fibrillation. These studies suggest that atrial fibrillation is a key contributor to frailty in elderly patients with type II diabetes. Based on this, in routine nursing care, the elderly patients' cardiopulmonary function can be improved by medication and increased exercise, thus reducing the impact of atrial fibrillation on their bodies.

The article "Study on Influencing Factors of Frailty in Elderly Patients with Type II Diabetes" was retracted in 2023. Reason: concerns about the peer review.

## 6. Conclusion

In conclusion, there is a close association between the degree of frailty in elderly patients with type II diabetes and exercise tolerance, exercise capacity, atrial fibrillation, anemia, and other hematologic diseases; therefore, in clinical nursing care, more attention paid to these aspects can improve the prevention and control efficiency for the treatment of this disease and avoid the occurrence of adverse events. In addition, gradually increasing the amount of exercise in elderly patients and strengthening their exercise capacity can improve heart systolic and diastolic function and blood circulation, thereby effectively relieving frailty. Our research needs more experimental samples to find the relationship with more blood diseases. Our experiment has limitations in this regard.

## Figures and Tables

**Table 1:** Patients' general information.

General information	
Age (years old)	60∼95
Average age (years old)	75.77 ± 8.22
Male-female ratio	155 : 177
Han to minority ratio	315 : 17
Proportion of patients receiving below junior high school education	89.76%
Proportion of manual workers	50.90%
Proportion of patients with an average monthly income above 2000 yuan	90.10%

**Table 2:** Univariate analysis of frailty in age and living habits.

Factors		Degree of frailty		
		Grade I	Grade II	Grade III
Age (years old)	60–65	16 (45.71%)	7 (20%)	12( 34.29%)
	66–70	26 (37.14%)	18 (25.71%)	26 (37.14%)
	71–75	15 (25.86%)	14 (24.14%)	29 (50%)
	76–80	17 (20%)	22 (25.88%)	46 (54.12%)
	80–85	7 (16.28%)	10(23.26%)	26 (60.47%)
	≥86	2 (4.88%)	14 (34.15%)	25 (60.98%)
	Total			
	*χ* ^2^		27.00	
	*P*		<0.01	

Dietary habits	Good	54 (26.73%)	63 (31.19%)	85 (42.08%)
	Poor	29 (22.31%)	22 (16.92%)	79 (60.77%)
	*χ* ^2^		12.50	
	*P*		<0.01	

Types of medication taking	0	0 (0.00%)	1 (100.00%)	0 (0.00%)
	1	28 (49.12%)	16 (28.07%)	13 (22.81%)
	2	45 (22.17%)	51 (25.12%)	107 (52.71%)
	3	9 (14.06%)	17 (26.56%)	38 (59.38%)
	4	1(14.29%)	0 (0.00%)	6 (85.71%)
	*χ* ^2^		33.95	
	*P*		<0.01	

Dislike for exercise	Yes	81 (27.27%)	75 (25.25%)	141 (47.47%)
	No	2 (5.71%)	10 (28.57%)	23 (65.71%)
	*χ* ^2^		8.06	
	*P*		<0.05	

**Table 3:** Univariate analysis of frailty in physique.

Factors		Degree of frailty				
		Grade I		Grade II		Grade III
Decreased exercise tolerance	Yes	53 (60.92%)	19 (21.84%)		15 (17.24%)	
	No	30 (12.24%)	66 (26.94%)		149 (60.82%)	
	*χ* ^2^		86.17			
	*P*		<0.01			

Reduced exercise capacity	Yes	67 (57.26%)	35 (29.91%)		15 (12.82%)	
	No	16 (7.44%)	50 (23.26%)		149 (69.3%)	
	*χ* ^2^		125.48			
	*P*		<0.01			

Body balance	Good	75 (38.07%)	57 (28.93%)		65 (32.99%)	
	Poor	8(5.93%)	28(20.74%)		99 (73.33%)	
	*χ* ^2^		61.60			
	*P*		<0.01			

Weakened coordination ability	Yes	69 (34.5%)	62 (31%)		69 (34.5%)	
	No	14 (10.61%)	23 (17.42%)		95 (71.97%)	
	*χ*2		46.48			
	*P*		<0.01			

Urinary incontinence	Yes	83 (25.86%)	84 (26.17%)		154 (47.98%)	
	No	0 (0%)	1 (9.09%)		10 (90.91%)	
	*χ*2		8.02			
	*P*		<0.05			

Anxiety	Yes	72 (31.72%)	51 (22.47%)		104 (45.81%)	
	No	11 (10.48%)	34 (32.38%)		60 (57.14%)	
	*χ*2		17.58			
	*P*		<0.01			

The article "Study on Influencing Factors of Frailty in Elderly Patients with Type II Diabetes" was retracted in 2023. Reason: concerns about the peer review.

**Table 4:** Univariate analysis of frailty in cardiovascular diseases.

Coronary heart disease				Heart failure			Atrial fibrillation		
Degree of frailty	Grade I	Grade II	Grade III	Grade I	Grade II	Grade III	Grade I	Grade II	Grade III
Yes	37 (37.76%)	31 (31.63%)	30 (30.61%)	78 (26.44%)	81 (27.46%)	136 (46.1%)	79 (26.87%)	80 (27.21%)	135 (45.92%)
No	46 (19.66%)	54 (23.08%)	134 (57.26%)	5 (13.51%)	4 (10.81%)	28 (75.68%)	4 (10.53%)	5 (13.16%)	29 (76.32%)
*χ* ^2^		20.96			11.58			12.49	
*P*		<0.01			<0.01			<0.01	

**Table 5:** Univariate analysis of frailty in other related diseases.

Pulmonary disease				Osteoarticular diseases			Anemia and other blood diseases		
Degree of frailty	Grade I	Grade II	Grade III	Grade I	Grade II	Grade III	Grade I	Grade II	Grade III
Yes	71 (29.34%)	63 (26.03%)	108 (44.63%)	78 (27.18%)	74 (25.78%)	135 (47.04%)	75 (28.3%)	69 (26.04%)	121 (45.66%)
No	12 (13.33%)	22 (24.44%)	56 (62.22%)	5 (11.11%)	11 (24.44%)	29 (64.44%)	8 (11.94%)	16 (23.88%)	43 (64.18%)
*χ* ^2^		10.90			6.43			9.54	
*P*		<0.01			<0.05			<0.05	

**Table 6:** Multiple logistic regression analyses of the influencing factors of frailty in elderly patients with type II diabetes.

Factors	B	Standard error	Wald*χ*^2^	Degree of freedom	Significance level	OR	Confidence interval 95%	
							Lower limit value	Upper limit value
Reduced exercise tolerance	1.59	0.53	9.05	1.00	0.00	4.91	1.74	13.84
Weakened exercise capacity	2.56	0.52	24.54	1.00	0.00	12.92	4.70	35.57
Anemia and other blood diseases	1.45	0.58	6.26	1.00	0.01	4.28	1.37	13.39
Atrial fibrillation	1.64	0.81	4.05	1.00	0.04	5.13	1.04	25.26

## Data Availability

The datasets used and/or analyzed during the current study are available from the corresponding author on reasonable request.
